The article "Porcine Fibrin Sealant Promotes Skin Wound Healing in Rats" was retracted in 2023. Reasons: signs of a paper mill; suspected computer-generated content; unreliable results or conclusions; concerns about the data.

# Porcine Fibrin Sealant Promotes Skin Wound Healing in Rats

**DOI:** 10.1155/2022/5063625

**Published:** 2022-06-23

**Authors:** Lihuo Zhang, Lu Liu, Jundong Zhang, Ping Zhou

**Affiliations:** ^1^State Key Laboratory of Molecular Engineering of Polymers, Department of Macromolecular Science, Fudan University, Shanghai 200433, China; ^2^Shanghai Haohai Biotechnology Co.Ltd., Shanghai 201613, China

## Abstract

**Objective:**

Fibrin sealant (FS) is widely used for skin wound healing, but data on porcine FS (PFS), a new type of FS, are limited. This study investigated the effects and potential mechanisms of porcine fibrin sealant (PFS) on skin wound healing in rats*. Methods*. Traumatic rats were randomly divided into three groups: control, PFS, and medical Vaseline. The wound area and wound index of the rats were measured within 14 days after surgery. Hematoxylin-eosin (H&E) staining and Masson staining were used to observe the pathological images and collagen formation on the wounded skin, respectively. To investigate the healing mechanisms, the enzyme-linked immunosorbent assay (ELISA) was used to detect platelet endothelial cell adhesion molecule-1 (CD31) and cluster of differentiation 34 (CD34) expression in the wounded skin. Additionally, quantitative real-time PCR (qRT-PCR) was used to evaluate the mRNA levels of the vascular endothelial growth factor (VEGF), fibroblast growth factor (FGF), and epidermal growth factor (EGF), and transforming growth factor-*β*1 (TGF-*β*1). Meanwhile, TGF-*β*1 protein expression was assessed by Western blot analysis.

**Results:**

Compared with the control group, both PFS and medical Vaseline treatment significantly reduced the wounded area and increased the wound closure rate. H&E staining showed that the cells in the PFS group proliferated rapidly, and the epidermis and dermis were thickened to some extent with a clear epidermal cell structure. Moreover, PFS promoted the formation of collagen and significantly increased the levels of CD31 and CD34 and the growth factors in the skin tissues of the traumatic rats.

**Conclusion:**

PFS effectively promoted skin wound healing, especially in tissue formation, reepithelialization, angiogenesis, and collagen deposition, in traumatic rat models. This study provides a new strategy and scientific foundation for PFS application in skin wound healing.

## 1. Introduction

As a vital organ of the human body, under normal state, the skin can reflect the health and stability of the body [1]. It has crucial physiological functions such as acting as a protective barrier, regulating the body temperature, and preventing loss of tissue fluid to maintain homeostasis [2]. Unfortunately, several factors, including trauma, inflammation, and burns, can cause skin wounds while performing daily chores [3]. In diabetic people with serious skin defects, their skin needs a longer healing time, and generally, longer healing time could lead to poorer outcomes [4, 5]. However, the healing of wounded skin is a complex process that involves a series of different cells and molecules, such as the various cytokines and growth factors released by the blood vessels, the migration and proliferation of epithelial cells, and the deposition and remodeling of extracellular matrix [6–9]. Even though wound healing is a challenging process due to the complex underlying biological processes, identification of effective treatments for skin wound repair is urgently needed. Thus, many researchers are focusing on investigating strategies that can promote wound closure and reduce wound index during healing.

The article "Porcine Fibrin Sealant Promotes Skin Wound Healing in Rats" was retracted in 2023. Reasons: signs of a paper mill; suspected computer-generated content; unreliable results or conclusions; concerns about the data.

Fibrin sealant (FS) is a biological adhesive containing fibrinogen and thrombin as its main components [10] and is widely used for skin wound healing [11, 12]. Due to its superior biocompatibility and biodegradability, FS can hardly cause inflammation, foreign body reaction, tissue necrosis, or extensive fibrosis. Conversely, FS can effectively promote the growth and formation of blood vessels, prevent tissue adhesion, and stop bleeding [13]. Overall, FS is an appropriate agent for healing skin wounds and has been widely used in various clinical fields. Portes et al. showed that FS could promote fibrin production in porcine vocal folds and contribute to wound healing [14]. Porcine FS (PFS) is a new biological hemostatic material made by extracting protein from porcine blood and is primarily composed of fibrinogen, thrombin, factor XIII, and calcium ion [15]. Wang et al. reported that promoting ulcer healing without an increase in bleeding could be achieved by a wound microvascular protective hemostatic technique consisting of PFS and conservative electrocoagulation [16]. However, there is no literature describing the effects of PFS on skin incisions.

In this study, we investigated the efficacy of PFS in incision healing and wound histomorphology in a traumatic rat model to assess its potential clinical applicability.

## 2. Materials and Methods

### 2.1. Experimental Animals

Thirty male SD rats of weight 180–220 g maintained under SPF conditions were randomly divided into three different groups: control, Vaseline (positive control), and PFS groups (*n* = 10 in each group). The animal experiments described in this study were authorized by the Experimental Animal Ethics Committee of Guangdong Medical Experimental Center (2022-0315).

Skin wounds were established based on previously described methods by Kanyu et al. [17]. Briefly, the rats were weighed and anesthetized by intraperitoneal injection of 10% pentobarbital sodium (0.3 g/kg). Their dorsal areas were thoroughly shaved and fixed in the prone position. Routine disinfection of the surgical site was performed, and surgical drapes were placed. Then, a full-thickness circular skin incision, 1.0 cm in diameter that extended to the muscular layer, was made on their back, and thereafter, the wound was kept dry.

The article "Porcine Fibrin Sealant Promotes Skin Wound Healing in Rats" was retracted in 2023. Reasons: signs of a paper mill; suspected computer-generated content; unreliable results or conclusions; concerns about the data.

The wounded skin of rats of the Vaseline and PFS groups were applied with medical Vaseline (Nanchang Baiyun Pharmaceutical Co., Ltd., China) and PFS (Shanghai Haohai Biotechnology Co., Ltd., China), respectively. In contrast, no treatment was performed on the wound of the control group. A Tegaderm film was used to cover all wounds for protection and was changed regularly every 3 days. The wound area of the rats was recorded on the 0, 3rd, 7th, 10th, and 14th day after surgery. Their wound index was recorded on the 3rd, 7th, 10th, and 14th day after surgery. The rats were sacrificed after 7 days and 14 days to extract the skin tissues of their wounds for the subsequent detection and analysis of other indicators.

### 2.2. Determination of Wound Area and Healing Rate

On the 3rd, 7th, 10th, and 14th day after excision surgery, the residual wound edge was drawn on the membrane, and the membrane was scanned for imaging to determine the wound area and healing rate. Image acquisition and calculation of the wound area were performed using the Image-J software. The healing rate was calculated using the following equation [18]:

(1) $$\begin{array}{c} H_{t}=\frac{\left(S_{0}-S_{t}\right)}{S_{0}}\times 100\%, \end{array}$$

where *H*_*t*_ represents the wound healing rate at time *t* after surgery, *S*_0_ represents the initial wound area, and *S*_*t*_ represents the wound healing area at time *t*.

### 2.3. Determination of Wound Index

The wound index of rats was recorded on the 3rd, 7th, 10th, and 14th day using the wound index scoring system. The wounds were scored by 3 different professionals following the scoring standard. The scoring criteria were based on the methods described by Patil et al. [19], which were as follows: 4 points suggested purulent necrosis; 3 points suggested that repair had not yet started, but the surrounding environment was healthy; 2 points suggested delayed but healthy healing; 1 point suggested incomplete but healthy healing; and 0 point suggested complete healing.

### 2.4. Hematoxylin-Eosin (H&E) Staining and Masson Staining

On completion of the separation of the rat skin tissues, a part of the tissue was fixed in formalin solution, followed by embedding and sectioning steps. Finally, H&E staining and Masson staining were performed on the skin tissues according to the procedure previously described by Lin [20] to show the wound tissues' changes and degree of collagen deposition.

The article "Porcine Fibrin Sealant Promotes Skin Wound Healing in Rats" was retracted in 2023. Reasons: signs of a paper mill; suspected computer-generated content; unreliable results or conclusions; concerns about the data.

### 2.5. Enzyme-Linked Immunosorbent Assay (ELISA)

The skin tissues of the wounds were taken from rats of each group and thoroughly grounded in prechilled PBS. The resulting homogenate was then centrifuged, and the supernatant was collected to detect CD31 and CD34 expressions in the skin tissues in strict accordance with the instructions of the ELISA Kit (Nanjing Jiancheng Bioengineering Institute, China).

### 2.6. Quantitative Real-Time PCR (qRT-PCR)

Total RNA of skin tissues was extracted using the total RNA extraction kit and reverse transcribed into cDNA following the manufacturer's instructions (Takara, Japan). cDNA underwent multiple reactions, following the protocol for qRT-PCR, using the following steps: 95 C for 1 min; 35 cycles of 95 C for 40 s, 58 C for 40 s, 72 C for 45 s, and 72 C for 10 min. The relative expression of genes was analyzed with the 2^−ΔΔCt^ method [21]. The primers used for qRT-PCR are given in Table 1.

### 2.7. Western Blot Analysis

The proteins were extracted from the tissues, quantified, and separated by 12% SDS-PAGE. Subsequently, the proteins were transferred to PVDF membranes, followed by a 1-hour blocking step using 5% nonfat dry milk at ambient temperature. Then, the membranes were incubated overnight at 4 C with the transforming growth factor-beta 1 (TGF-*β*1) primary antibody (ab215715, Abcam, UK) and GAPDH (ab8245, Abcam). Next, they were rinsed with TBST and incubated with secondary antibody (ab150077, Abcam) at ambient temperature for 1 hour, followed by rinsing. Finally, a chemiluminescence reagent was added to develop the protein, and the Image-J software was used to analyze the gray values of the protein bands. The relative protein expression was calculated using the GAPDH as an internal reference.

### 2.8. Statistical Analysis

The SPSS (version 21.0) was used for statistical analyses. For comparisons between the groups, the *t*-test was used. The one-way analysis of variance was used for pairwise comparison among different groups. Experimental data were expressed as mean ± standard deviation (SD). A difference was considered statistically significant for *p* < 0.05.

## 3. Results

### 3.1. PFS Promotes Skin Wound Healing in Rats

We investigated the effect of PFS on the wounds of rats by measuring their wound area. On the 3rd, 7th, 10th, and 14th day, the wound area of the rats in all three groups gradually decreased, and the wound closure rate was significantly increased. However, on the 3rd, 7th, and 10th day, rats from the PFS group had smaller wound areas and faster wound closure rate compared to those from the control group (*p* < 0.01), as shown in Figures 1(a)–1(c).

The article "Porcine Fibrin Sealant Promotes Skin Wound Healing in Rats" was retracted in 2023. Reasons: signs of a paper mill; suspected computer-generated content; unreliable results or conclusions; concerns about the data.

### 3.2. Impact of PFS on the Skin Wound Index of Rats

As recorded on the 3rd, 7th, 10th, and 14th day after surgery, the wound index of rats in the three groups gradually decreased with time. As shown in Figure 2, the PFS group had a significantly lower wound index than the Vaseline group (*p* < 0.05). However, although the wound index of the Vaseline group was lower than that of the control group, the difference was not statistically significant (*p* > 0.05).

### 3.3. Effect of PFS on the Histomorphology and Collagen Deposition in the Wounded Skin of Rats

Figure 3(a) shows the H&E staining results of the control group and distinct characteristics such as infiltration of various inflammatory cells, slow formation of granulation tissue, and few collagen fibers and epidermal cells, and a low degree of epithelialization could be observed. In contrast, the Vaseline group had lesser inflammatory cell infiltration. Additionally, the Vaseline group had granulation of tissues, their collagen fibers were more neatly arranged, and they had markedly increased degree of epithelialization. Interestingly, the PFS group displayed significant cell proliferation, thickened epidermis and dermis, clear structure of epidermal cells, reduced inflammatory cells, and more granulation tissue. Furthermore, a greater amount of collagen could be observed and was more neatly arranged in the PFS group, as shown in Figure 3(b). According to Masson staining results, in comparison with the Vaseline group, a marked increase in collagen formation was found in the PFS group (*p* < 0.01). Although the collagen formation of the Vaseline group was greater than the control group, the difference was not statistically significant (*p* > 0.05), as shown in Figures 3(b) and 3(c).

### 3.4. Effect of PFS on Angiogenesis in the Wounded Skin of Rats

CD31 and CD34 proteins are important endothelial cell markers [22] that can represent the degree of tissue vascularization to a certain extent. ELISA assay on the rats' skin tissues confirmed that in comparison with the Vaseline group, significantly higher levels of CD31 and CD34 were found in the PFS group on the 7th day after surgery (*p* < 0.01). However, no marked differences were found in CD31 and CD34 expression levels between the control and Vaseline groups (*P* > 0.05, Figures 4(a) and 4(b)).

In addition, VEGF, FGF, and EGF can effectively promote endothelial cell proliferation and, consequently, angiogenesis [23]. The results of qRT-PCR shown in Figures 4(c) and 4(d) showed that the mRNA expression of VEGF, FGF, and EGF in the wounded skin of the PFS group was significantly increased compared with that of the Vaseline group on the 7th and 14th day after surgery (*p* < 0.01). Collectively, PFS can significantly promote the neovascularization of injured skin in rats via increasing the mRNA expression of VEGF, FGF, and EGF.

The article "Porcine Fibrin Sealant Promotes Skin Wound Healing in Rats" was retracted in 2023. Reasons: signs of a paper mill; suspected computer-generated content; unreliable results or conclusions; concerns about the data.

### 3.5. Effect of PFS on TGF-*β*1 Expression in the Wounded Skin of Rats

TGF-*β* can effectively mediate new collagen formation and promote angiogenesis [24]. As shown in Figure 5, the expression of both TGF-*β*1 mRNA and protein in the skin tissues of the PFS group was higher than that of the Vaseline group on the 7th and 14th day after surgery (*p* < 0.01). Compared with the control group, the Vaseline group exhibited a significantly increased expression of TGF-*β*1 mRNA and protein in the wounded skin tissues on the 7th day, and the level of TGF-*β*1 protein was markedly increased on the 14th day after surgery.

## 4. Discussion

Wound healing is a complex process involving epidermal reepithelialization, angiogenesis, and collagen deposition [23]. Keratinocytes, monocytes, and macrophages play an important role in regulating epidermal reepithelialization, and this process is mainly associated with EGF [25], VEGF, and FGF production [26], which induce cell migration, proliferation, and matrix formation [27]. Collagen deposition is one of the test criteria for partial dermal repair, and collagen formation can effectively promote wound healing, but excessive deposition can disrupt the balance between collagen deposition and degradation and ultimately lead to hypertrophic scarring [28, 29]. FS is a natural hydrogel. It is the end product of the physiological blood coagulation cascade, directly involved in wound healing, and plays overlapping roles in wound healing by mediating both hemostasis and homeostasis [30]. Rapid hemostasis and effective wound closure are very important in wound repair because delays could lead to increasing risks of complications.

In recent years, several medical adhesives have been researched to improve wound healing. In a study by Canonico, the author investigated the use of human fibrin glue in surgical operations and found that it was effective in preventing local hemorrhagic complications and concurrent coagulation disorders [31]. Platelet gel (PG) has been used in combination to promote the healing of recalcitrant lower extremity ulcers [32]. Although no recurrence of ulcers and no adverse reactions were observed with PG, there was no control group to validate these findings. Recently, there have been renewed interests in active leptospermum honey dressings as an approach to wound management due to their antimicrobial and immunological effects and adhesive or sealant properties [33, 34]. However, these studies have mostly been investigational, with a small sample size and no control group. Furthermore, higher levels of evidence from clinical trials are needed before any practice recommendations can be made. In this study, PFS was implemented because it is a new type of FS that has been shown to have superior properties compared with commonly used FS [35]. Its use has been associated with a lesser risk of blood-borne disease or virus infections compared with FS [35, 36]. Considering that PFS is widely used in clinical surgery for hemostasis and studies regarding its applicability in wound healing are limited, in this study, the potential of PFS in wound healing was compared to a control and Vaseline group. We found that PFS could significantly reduce the wound area and improve the wound closure rate with a gradual decrease in the wound index in rats. In addition, PFS markedly reduced the infiltration of various inflammatory cells in the wounded skin tissue and promoted angiogenesis and collagen formation, thereby stimulating wound healing in rats.

The article "Porcine Fibrin Sealant Promotes Skin Wound Healing in Rats" was retracted in 2023. Reasons: signs of a paper mill; suspected computer-generated content; unreliable results or conclusions; concerns about the data.

Endothelial progenitor cells (EPCs) are a specialized class of stem cells that can actively participate in the proliferation of endothelial cells and can differentiate into vascular endothelial cells. CD31 and CD34 are currently considered as important markers of EPCs, and both are involved in angiogenesis during the embryonic period and have a pivotal role in regulating postnatal physiological and pathological angiogenesis [37]. In this present study, the results showed that PFS significantly increased the levels of CD31 and CD34, which indicated that PFS could promote angiogenesis and thereby improve wound healing.

EGF is mainly synthesized and secreted by platelets and damaged keratinocytes, promoting cell division. EGF can substantially stimulate the division and proliferation of various cells, such as keratinocytes and fibroblasts, and also accelerate protein synthesis in the tissue repair cells, epithelialization of wounds, and ultimately complete wound healing [38, 39]. VEGF can exhibit a variety of biological activities that can markedly enhance microvascular permeability, promote proliferation and the migration of endothelial cells and macrophages, and thereby induce the expression of interstitial collagenase [40]. Moreover, VEGF has been found to be responsible for promoting wound healing, tissue repair, and tissue regeneration. During the skin wound healing process, blood vessels provide nutrients and eliminate metabolic wastes from the wounds at the early stage. Then, the formation of a large number of new blood vessels supplies additional nutrients during the proliferation phase. For example, VEGF alone can normalize wound healing in diabetic animal models [41]. FGF is a group of active polypeptides present in organisms and expressed in various tissues and cells. FGF can promote mitosis of epithelial cells and the migration of fibroblasts and endothelial cells to the wounded site and substantially enhance angiogenesis. A number of previous studies have shown that FGF expression is increased at the wounded site [42] and can effectively accelerate skin and epidermal repair [43]. Fibroblasts, the most common cells found in connective tissues, play a key role during skin wound healing, particularly during the proliferation and remodeling phases. Specifically, during wound healing, the fibroblasts play an important role in maintaining the physical integrity of connective tissue, participating in wound closure, and producing and remodeling the extracellular matrix. FGF can also promote the formation of collagenase, thus accelerating collagen degradation and reducing the formation of scars [44]. In this study, after the application of PFS to the skin wounds of rats, a significant increase in the expression levels of VEGF, FGF, and EGF was found, suggesting that PFS can promote the expression of growth factors, cell migration, proliferation, and neovascularization, resulting in the better wound repair than other two groups. However, more research studies are needed to confirm these findings.

The article "Porcine Fibrin Sealant Promotes Skin Wound Healing in Rats" was retracted in 2023. Reasons: signs of a paper mill; suspected computer-generated content; unreliable results or conclusions; concerns about the data.

TGF-*β* is an antifibrotic cytokine, and its high expression can effectively contribute to rapid healing in the early stage of an injury and has also been closely associated with wound contraction, cicatricial contracture, and collagen formation [45, 46]. In this present study, both qRT-PCR and Western blot results showed that TGF-*β*1 expression was markedly upregulated in the PFS group and could thereby effectively promote the formation of collagen. These findings were consistent with the results of Masson staining and could be among the possible mechanisms via which PFS significantly promoted skin wound healing in rats.

## 5. Conclusion

In summary, PFS could significantly reduce the wound area of rats, improve their wound closure rate, and promote neovascularization and collagen formation. These results suggest PFS as an effective agent in wound healing and with promising clinical values. The therapeutic mechanism of action of PFS could be related to TGF-*β*1, but the specific mechanism needs to be further investigated.

## Figures and Tables

**Figure 1:** Effect of PFS on rat skin wound area and healing rate. (a) Images of rat wound area at indicated time. (b) Statistical analysis of rat wound area at indicated time. (c) Statistical analysis of rat wound healing rate at indicated time. ^*∗∗*^*P* < 0.01 vs. the control group, *n* = 5.

The article "Porcine Fibrin Sealant Promotes Skin Wound Healing in Rats" was retracted in 2023. Reasons: signs of a paper mill; suspected computer-generated content; unreliable results or conclusions; concerns about the data.

**Figure 2:** Effect of PFS on rat wound index. ^*∗*^*P* < 0.05 and ^*∗∗*^*p* < 0.01 vs. the Vaseline group, *n* = 5.

**Figure 3:** Effect of PFS on histomorphology and collagen deposition of the wounded skin of rats on the 14^th^ day. (a) H&E staining-based detection for the pathological histomorphology of the wounded skin. (b) Masson staining detection for collagen formation in the wounded skin of rats. (c) Collagen volume fraction of the wounded skin in rats. ^*∗∗*^*P* < 0.01 vs. the Vaseline group, *n* = 5.

**Figure 4:** Effect of PFS on the protein expression of CD31 (a) and CD34 (b). Effect of PFS on the mRNA expression of VEGF, FGF, and EGF on the 7th (c) and 14th (d) day after surgery. ^*∗∗*^*P* < 0.01, ^*∗∗∗*^*p* < 0.001, *n* = 5.

**Figure 5:** Effect of PFS on TGF-*β*1 expression in rat wounded skin. (a) qRT-PCR-based detection for TGF-*β*1 mRNA expression. (b) Western blot-based detection for TGF-*β*1 protein expression. ^*∗∗*^*P* < 0.01, ^*∗∗∗*^*p* < 0.001, *n* = 5.

**Table 1:** The primers used for qRT-PCR.

Gene	Sequences (5′-3′)	

VEGF	Forward	GACACACCCACCCACATACA
	Reverse	ACATCCTCCTCCCAACTCAA

FGF	Forward	CTGTCTCCCGCACCCTATC
	Reverse	CTTTCTCCCTTCCTGCCTTT

EGF	Forward	CCCGTGTTCTTCTGAGTTCC
	Reverse	TGTAACCGTGGCTTCCTTCT

TGF-*β*1	Forward	CGCAATCTATGACAAAACCAAA
	Reverse	ACAGCCACTCAGGCGTATC

*β*-Actin	Forward	GGGTTACGCGCTCCCTCAT
	Reverse	GTCACGCACGATTTCCCTCTC

## Data Availability

The data used to support the findings of this study are available from the corresponding author upon request.

## References

[1] Khodaii Z., Afrasiabi S., Hashemi S. A., Ardeshirylajimi A., Natanzi M. M. (2019). Accelerated wound healing process in rat by probiotic Lactobacillus reuteri derived ointment. *Journal of Basic and Clinical Physiology and Pharmacology*.

[2] Reis M. B., Pereira P. A. T., Caetano G. F. (2017). Lipoxin A4 encapsulated in PLGA microparticles accelerates wound healing of skin ulcers. *PLoS One*.

[3] Browne S., Pandit A. (2015). Biomaterial-mediated modification of the local inflammatory environment. *Frontiers in Bioengineering and Biotechnology*.

[4] Chin J. S., Madden L., Chew S. Y., Becker D. L. (2019). Drug therapies and delivery mechanisms to treat perturbed skin wound healing. *Advanced Drug Delivery Reviews*.

[5] Xu W.-K., Tang J.-Y., Yuan Z. (2019). Accelerated cutaneous wound healing using an injectable teicoplanin-loaded PLGA-PEG-PLGA thermogel dressing. *Chinese Journal of Polymer Science*.

The article "Porcine Fibrin Sealant Promotes Skin Wound Healing in Rats" was retracted in 2023. Reasons: signs of a paper mill; suspected computer-generated content; unreliable results or conclusions; concerns about the data.

[6] Singer A. J., Clark R. A. (1999). Cutaneous wound healing. *New England Journal of Medicine*.

[7] Kim B. J., Cheong H., Choi E.-S. (2017). Accelerated skin wound healing using electrospun nanofibrous mats blended with mussel adhesive protein and polycaprolactone. *Journal of Biomedical Materials Research Part A*.

[8] Aragão-Neto A. C., Soares P. A. G., Lima-Ribeiro M. H. M., Carvalho E. J. A., Correia M. T. S., Carneiro-da-Cunha M. G. (2017). Combined therapy using low level laser and chitosan-policaju hydrogel for wound healing. *International Journal of Biological Macromolecules*.

[9] Jeon E. Y., Hwang B. H., Yang Y. J. (2015). Rapidly light-activated surgical protein glue inspired by mussel adhesion and insect structural crosslinking. *Biomaterials*.

[10] Gao Y. H., Chen Z. H., Guo H. L. (2014). Effect of fibrin glue on healing of canine skin incisions. *Progress in Veterinary Medicine*.

[11] Park J. H., Choi S. H., Park S. J. (2017). Promoting wound healing using low molecular weight fucoidan in a full-thickness dermal excision rat model. *Marine Drugs*.

[12] Banitt M., Malta J. B., Soong H. K., Musch D. C., Mian S. I. (2009). Wound integrity of clear corneal incisions closed with fibrin and N-butyl-2-cyanoacrylate adhesives. *Current Eye Research*.

[13] Guo S., Liu H., Zhou M. M. (2016). Research progress of medical fibrin sealant. *China Pharmacy*.

[14] Portes K. P., de Campos Duprat A., Lancellotti C. L. P., Silva L., de Souza F. C. (2012). Influence of selant fibrin on the wound healing of the pigs vocal folds. *Brazilian Journal of Otorhinolaryngology*.

[15] Wu Q. R. (2019). *Study on the Prescription of Porcine Fibrinogen Freeze-Dried Preparation and its Freeze-Drying Process*.

[16] Wang J., Wu Q., Yan Y. (2020). Effectiveness of fibrin sealant as hemostatic technique in accelerating ESD-induced ulcer healing: a retrospective study. *Surgical Endoscopy*.

[17] Kan Y. (2019). *Moxibustion Enhances Wound Healing in Traumatic Rats and its Underlying Mechanism*.

[18] Ou S. L., Chen Z. M., Wu Q. R. (2018). Effects of porcine fibrin sealant on the healing of wounds and hydroxyproline expression in rats. *Science Technology and Engineering*.

[19] Patil M. V. K., Kandhare A. D., Bhise S. D. (2012). Pharmacological evaluation of ethanolic extract of Daucus carota Linn root formulated cream on wound healing using excision and incision wound model. *Asian Pacific Journal of Tropical Biomedicine*.

[20] Lin Q. M. (2020). *The Study of Chinese Medicine Prescription BaiJinfeng for Skin Wound Repair*.

[21] Yang J., Chen Z., Pan D., Li H., Shen J. (2020). Umbilical cord-derived mesenchymal stem cell-derived exosomes combined pluronic F127 hydrogel promote chronic diabetic wound healing and complete skin regeneration. *International Journal of Nanomedicine*.

The article "Porcine Fibrin Sealant Promotes Skin Wound Healing in Rats" was retracted in 2023. Reasons: signs of a paper mill; suspected computer-generated content; unreliable results or conclusions; concerns about the data.

[22] Lionello M., Staffieri A., Marioni G. (2012). Potential prognostic and therapeutic role for angiogenesis markers in laryngeal carcinoma. *Acta Oto-Laryngologica*.

[23] Barrientos S., Stojadinovic O., Golinko M. S., Brem H., Tomic-Canic M. (2008). Perspective article: growth factors and cytokines in wound healing. *Wound Repair and Regeneration*.

[24] Eppley B. L., Woodell J. E., Higgins J. (2004). Platelet quantification and growth factor analysis from platelet-rich plasma: implications for wound healing. *Plastic and Reconstructive Surgery*.

[25] Sant’Ana E. M. C., Gouvêa C. M. C. P., Durigan J. L. Q., Cominetti M. R., Pimentel E. R., Selistre-de-Araújo H. S. (2011). Rat skin wound healing induced by alternagin-C, a disintegrin-like, Cys-rich protein from Bothrops alternatus venom. *International Wound Journal*.

[26] Smith A. M., Moxon S., Morris G. A. (2016). Biopolymers as wound healing materials. *Wound Healing Biomaterials*.

[27] Sun B. K., Siprashvili Z., Khavari P. A. (2014). Advances in skin grafting and treatment of cutaneous wounds. *Science*.

[28] Dabiri G., Campaner A., Morgan J. R., Van De Water L. (2006). A TGF-*β*1-dependent autocrine loop regulates the structure of focal adhesions in hypertrophic scar fibroblasts. *Journal of Investigative Dermatology*.

[29] Zhu Z., Ding J., Shankowsky H. A., Tredget E. E. (2013). The molecular mechanism of hypertrophic scar. *Journal of Cell Communication and Signaling*.

[30] Heher P., Mühleder S., Mittermayr R., Redl H., Slezak P. (2018). Fibrin-based delivery strategies for acute and chronic wound healing. *Advanced Drug Delivery Reviews*.

[31] Canonico S. (2003). The use of human fibrin glue in the surgical operations. *Acta BioMedica*.

[32] Chen T. M., Tsai J.-C., Burnouf T. (2010). A novel technique combining platelet gel, skin graft, and fibrin glue for healing recalcitrant lower extremity ulcers. *Dermatologic Surgery*.

[33] Hamzaoglu İ., Saribeyoglu K., Durak H. (2000). Protective covering of surgical wounds with honey impedes tumor implantation. *Archives of Surgery*.

[34] Emsen I. M. (2007). A different and safe method of split thickness skin graft fixation: medical honey application. *Burns*.

[35] Roberts I. V., Bukhary D., Valdivieso C. Y. L., Tirelli N. (2020). Fibrin matrices as (injectable) biomaterials: formation, clinical use, and molecular engineering. *Macromolecular Bioscience*.

[36] Yang Y., Wang X., Zha K. (2021). Porcine fibrin sealant combined with autologous chondrocytes successfully promotes full‐thickness cartilage regeneration in a rabbit model. *Journal of Tissue Engineering and Regenerative Medicine*.

The article "Porcine Fibrin Sealant Promotes Skin Wound Healing in Rats" was retracted in 2023. Reasons: signs of a paper mill; suspected computer-generated content; unreliable results or conclusions; concerns about the data.

[37] Lin C. P., Lin F. Y., Huang P. H. (2013). Endothelial progenitor cell dysfunction in cardiovascular diseases: role of reactive oxygen species and inflammation. *BioMed Research International*.

[38] Gokakin A. K., Deveci K., Kurt A. (2013). The protective effects of sildenafil in acute lung injury in a rat model of severe scald burn: a biochemical and histopathological study. *Burns*.

[39] Tan N., Thode H. C., Singer A. J. (2014). The effect of controlled mild hypothermia on large scald burns in a resuscitated rat model. *Clinical and Experimental Emergency Medicine*.

[40] Elcin Y. M., Dixit V., Gitnick G. (2001). Extensive in vivo angiogenesis following controlled release of human vascular endothelial cell growth factor: implications for tissue engineering and wound healing. *Artificial Organs*.

[41] Galiano R. D., Tepper O. M., Pelo C. R. (2004). Topical vascular endothelial growth factor accelerates diabetic wound healing through increased angiogenesis and by mobilizing and recruiting bone marrow-derived cells. *American Journal of Pathology*.

[42] Akita S., Akino K., Imaizumi T., Hirano A. (2008). Basic fibroblast growth factor accelerates and improves second-degree burn wound healing. *Wound Repair and Regeneration*.

[43] Meduri A., Aragona P., Grenga P. L., Roszkowska A. M. (2012). Effect of basic fibroblast growth factor on corneal epithelial healing after photorefractive keratectomy. *Journal of Refractive Surgery*.

[44] Wang J., Ding J., Jiao H. (2011). Human hypertrophic scar-like nude mouse model: characterization of the molecular and cellular biology of the scar process. *Wound Repair and Regeneration*.

[45] Mokoena D., Dhilip Kumar S. S., Houreld N. N., Abrahamse H. (2018). Role of photobiomodulation on the activation of the Smad pathway via TGF-*β* in wound healing. *Journal of Photochemistry and Photobiology B: Biology*.

[46] Rezaii M., Oryan S., Javeri A. (2019). Curcumin nanoparticles incorporated collagen-chitosan scaffold promotes cutaneous wound healing through regulation of TGF-*β*1/Smad7 gene expression. *Materials Science and Engineering*.

